# Fabrication of a Lead Head Made of the Carbon-Fiber-Reinforced Composite for the Temporary Cardiac Pacemaker

**DOI:** 10.1155/2021/7507555

**Published:** 2021-09-23

**Authors:** Yucheng Zhou, Xuming Lin, Zhao Yang, Xiaotong Han, Meng Liu

**Affiliations:** ^1^Emergency Department, Hunan Provincial People's Hospital, The First-Affiliate Hospital of Hunan Normal University, Changsha, Hunan 410005, China; ^2^Electromyogram Department, Hunan Province Hospital of Chinese Medicine, The Second-Affiliate Hospital of Hunan University of Chinese Medicine, Changsha, Hunan 410005, China

## Abstract

Compared with traditional leads, carbon fiber composite leads have a series of advantages such as lightweight, soft texture, and high conductivity. In this experiment, we attempted to improve the existing carbon-fiber-based TTCP metal leads by using carbon-fiber-graphene-woven leads or conductive cloth, so as to solve a series of defects of TTCP metal leads commonly used in the clinical temporary cardiac pacemaker. We performed a series of measurements, including resistance comparisons and stability checks on the finished product characteristics. The results showed that the resistivity of the whole lead did not change significantly after modification, and the carbon fiber bundle was stable and easily deformed under lower stress to reduce the damage to the myocardium, which had excellent clinical application value.

## 1. Introduction

Temporary transvenous cardiac pacing (TTCP) is a potential life-saving intervention [1], primarily for the treatment of symptomatic tachycardia and the relief of various types of reversible symptomatic heart block [2, 3]. In addition, TTCP can be used as a bridge to permanent cardiac pacing when permanent pacing cannot be directed or immediately used or when certain conditions preclude implantation of a permanent pacemaker. Other possible indications include myocardial infarction and/or conduction system injury after cardiac surgery [4, 5].

Figure 1 shows the ultrasonic image of bleeding and thrombus caused by electrode insertion into the myocardium.  Figure 2 shows the CT image of the lead penetrating the interventricular septum. The specificity of the surgical operation often entails a series of complications with TTCP, which can be categorized into two main groups: venous access-related complications or pacemaker catheter-related complications. Ultrasound-guided venous access has been shown to be safe, whereas pacemaker lead-related complications are frequently seen in clinical practice [6]. The standard TTCP lead has no fixed mechanism, which has a blunt, smooth, stiff tip that is electrically stimulated by direct contact with the myocardium through the negative pole of the lead. In the clinical use of TTCP, due to the stiffness of its leads, the placement of pacing leads in the right ventricle often promotes ectopic ventricular activity, and occasionally prolonged ventricular arrhythmias have been observed. Even worse, the pacing lead may penetrate the ventricular wall and occasionally perforate, increasing the risk of death during hospitalization [1, 7–11]. Studies have shown that the incidence of heart perforation is 0.1–3% [4, 12, 13]. In clinical practice, the incidence of sudden cardiac death in patients with pacemaker lead perforation is between 12 and 31%.

Carbon fiber is a special type of fibrous material obtained by carbonizing and graphitizing organic fibers and combining adjacent carbon atoms into a planar network [14]. Carbon fiber materials usually contain more than 90% carbon [14, 15], and they have excellent properties such as high temperature resistance, wear resistance, high electrical conductivity, and corrosion resistance, as well as remarkable anisotropy, flexibility, and processability [16]. Carbon fiber material is a superhydrophobic material because it consists of inert carbon atoms, with almost no active functional groups on the surface and very low surface chemical activity [17].

In order to solve the problem of cardiac injury and even perforation caused by TTCP in clinical applications, we designed a flexible lead tip made of carbon fiber composite material to replace the rigid metal lead tip at the negative end of TTCP leads. According to the experimental requirements, the flexibility and outstanding electrical conductivity of the carbon fiber composite were utilized to greatly reduce the incidence of atrial and ventricular wall perforations caused by lead electrodes of temporary pacemakers without affecting the electrical stimulation effect of the pacemaker. In this experiment, the electrical conductivity and stability of the flexible tip of the modified anode lead were measured, and the resistivity of the flexible tip made of carbon fiber material was compared with that of the hard tip made of conventional metal material, and the feasibility of a pacemaker lead based on carbon fiber composites was analyzed.

## 2. Experimental Materials

### 2.1. Preparation of the Carbon Fiber Composite Bundle and Carbon Fiber Cloth

To obtain a diameter similar to that of conventional leads, we prepared a composite bundle of carbon fibers with a diameter of 0.8 mm by assembling 2400 carbon fiber filaments closely together.

The carbon fiber cloth was factory-produced. Carbon fiber strands containing 95% carbon were woven into a uniform carbon fiber cloth with a thickness of 0.8 to 1.2 mm, an average mass of 20 g/m^2^, and a square resistance of 30 Ω.

### 2.2. Experimental Design

#### 2.2.1. Modified by the Carbon Fiber Composite Bundle

The experiments were based on a common clinical temporary pacemaker lead, and an attempt was made to modify it with carbon fibers. In the experimental preparation, the insulating layer between the positive and negative electrodes of the original lead was firstly removed, and then the central conductive material was removed; the central conductive material was replaced by a carbon fiber bundle of the same length, and the two conductive materials were tightly connected and fixed with a conductive double-sided carbon tape to obtain a TTCP lead modified with a carbon fiber composite bundle.  Figure 3 shows the carbon fiber bundle-modified TTCP lead.

#### 2.2.2. Modified by Carbon Fiber Cloth

Take a pacemaker lead of the same type and remove the rigid metal contact head on the lead. Unlike using carbon fiber bundles, we drop the removal of the conductive metal in the center of the lead in this operation and, instead, wrap the carbon fiber cloth around the built-in metal lead while securing it with a conductive double-sided carbon tape, using the external conductive carbon fiber cloth as a buffer, to obtain a carbon fiber cloth-modified TTCP lead.  Figure 4 shows the carbon fiber cloth-modified TTCP lead.

## 3. Characteristics of Leads

### 3.1. Resistance Test

The resistance of the lead was measured with a digital contact resistance sorter (HPS2515) by intercepting 135 cm and 2 cm of the core of the carbon fiber heating lead, respectively, clamping the ends of this part with the digital contact resistance sorter test, and using the resistance measurement function to determine its resistance and calculate its resistivity. The resistance of the TTCP lead (total length: 135 cm) and TTCP lead modified with the carbon fiber (total length: 135 cm, of which the carbon fiber part is 2 cm) was measured by the same method of the digital contact resistance sorter, and their resistivity was calculated. The experiment was conducted at 25.0°C and 37.0°C to obtain the experimental data, respectively.

### 3.2. Stability Test

We also tested the physical stability of several modified leads. Simulated clinical surgery was performed under the same operating conditions, multiple leads were punctured and removed under external conditions, and the physical state was evaluated over time.

### 3.3. Softness Comparison

Three groups of leads of the same length were cut and tested for stress when bent at 90°. The value of the pressure may well reflect the external force applied to the bent lead [18, 19]. Through the measurement of this value, the flexibility of small electric leads and cables can be quantitatively characterized, and the maximum pressure of lead tips on the vessel wall and myocardium during TTCP is deduced.

## 4. Results and Discussion

The diameter of the carbon fiber lead is 0.8 mm, and the diameter of the temporary pacemaker TTCP lead is 0.4 mm, from which the cross-sectional area of the lead can be obtained, so the resistivity of the sample can be found by the following equation:

(1) $$\begin{array}{c} R=\rho \;\frac{L}{S}. \end{array}$$

In this equation, *R* is the resistance, Ω; *ρ* is the resistivity, Ω·m; *L* is the length, *m*; *S* is the cross-sectional area of the sample.

Table 1 shows that the resistivity of the carbon fiber lead is lower than that of the TTCP metal lead, indicating that the carbon fiber lead has excellent conductivity, and the conductivity of the TTCP lead improved with the carbon fiber is not theoretically reduced. Interestingly, after the carbon-fiber-modified TTCP lead was operated, the resistance of the carbon fiber bundle-modified lead increased slightly compared with the theoretical value. As to the carbon fiber cloth-modified lead, however, resistance doubled. The possible causes of this phenomenon were speculated: (i) the carbon fiber portion of the modified TTCP lead is connected to the original TTCP metal lead portion by direct contact, and this portion is not closely connected, resulting in increased resistance; (ii) the carbon fiber portion of the modified TTCP lead has a different lead cross-sectional diameter than the original TTCP metal lead portion, resulting in an increase in the total resistance of the lead. There was a gap between the carbon fiber monofilaments, which might lead to resistance measurement error. The resistance of the carbon fiber bundle-modified lead is changed from 6.60 Ω to 7.39 Ω, with little effect on the conductivity. Based on the available data, a subsequent TTCP catheter with excellent conductivity and uniform size was obtained with minor modifications.

In the stability experiments of several different modified filaments, we have found that compared with the existing TTCP on the market, carbon fiber filaments have higher physical stability. In a variety of external environments, the carbon fiber filament is not fractured or separated after repeated friction puncture, and the appearance and integrity of the filament are well maintained. For carbon fiber cloth-modified TTCP lead, due to the particularity of its preparation, after friction puncture, the surface of carbon fiber cloth was damaged, and the carbon fiber was broken and separated, suggesting that its physical stability was poor, which was not conducive to clinical applications.

Three sets of leads of the same length were taken and tested for the stresses when they were made to bend at 90°. From the measurement of this value, we observed a deformation of 90° for each group of leads under different stresses. The deformation of the conventional TTCP leads reached 90° when the force was 208.4 N at the cut length, while the force was 6.7 N (carbon fiber composite leads) and 120.3 N (carbon fiber fabric-modified TTCP leads) when the carbon-fiber-modified TTCP leads reached the same deformation angle, respectively. It can be roughly deduced that the pressure on the vessel wall, ventricular wall, and atrial wall can be reduced by 96.8% and 42.3%, respectively, for each group of leads during the procedure. This suggests that carbon fiber composite leads are also better than carbon fiber fabric-modified TTCP leads in terms of softness, which can greatly reduce the damage to the patient during the procedure. Taking all aspects into consideration, we found that the carbon fiber fabric-modified TTCP leads seemed to have better overall performance. Temporary cardiac pacing is very important for emergency medicine [20]. This work may benefit the temporary cardiac pacing technique, along with other techniques such as mathematical analysis [21–23] and nanotechnology [24, 25].

## 5. Conclusions

Temporary transvenous cardiac pacing is often used to resuscitate critically ill patients, and a soft conductive substitute material is needed to reduce the casualties caused by TTCP leads. According to our experiment, carbon fiber lead has better conductivity than TTCP metal lead, while carbon fiber material is light and soft and can deform under lower pressure, which plays a good role in protecting the myocardium. Using it as a temporary pacemaker electrode lead can greatly reduce the risk of atrial and ventricular wall perforation caused by TTCP electrode lead and improve the electrical conductivity. The lead made of the carbon fiber composite bundle is more stable and has better electrical conductivity than carbon fiber cloth. Therefore, pacemaker lead based on carbon fiber composite material is an excellent functional lead.

## Figures and Tables

**Figure 1:** Ultrasonic image of bleeding and thrombus caused by electrode insertion into the myocardium.

**Figure 2:** CT image of the lead penetrating the interventricular septum.

**Figure 3:** Carbon fiber bundle-modified TTCP lead.

**Figure 4:** Carbon fiber cloth-modified TTCP lead.

**Table 1:** Lead resistance measurement results.

Types of leads	25°C		37°C	
	Resistance (Ω)	Resistivity (Ω·m)	Resistance (Ω)	Resistivity (Ω·m)
Conventional TTCP lead (135 cm)	6.60	6.140 × 10^−7^	6.65	6.187 × 10^−7^
Carbon fiber lead (135 cm)	1.29	4.801 × 10^−7^	1.26	4.689 × 10^−7^
Carbon fiber lead (2 cm)	0.0191	4.801 × 10^−7^	0.0187	4.689 × 10^−7^
Carbon fiber bundle-modified TTCP lead (135 cm)	7.39	—	7.45	—
Carbon fiber cloth-modified TTCP lead (135 cm)	12.5	—	13.2	—

## Data Availability

The data used to support the findings of this study are included within the article.
